The article "Enterococcal Infective Endocarditis following Periodontal Disease in Dogs" was retracted in 2021. Reasons: errors in the methods; concerns about the data; concerns about the results or conclusions.

# Enterococcal Infective Endocarditis following Periodontal Disease in Dogs

**DOI:** 10.1371/journal.pone.0146860

**Published:** 2016-01-11

**Authors:** Teresa Semedo-Lemsaddek, Marta Tavares, Berta São Braz, Luís Tavares, Manuela Oliveira

**Affiliations:** Interdisciplinary Centre of Research in Animal Health (CIISA), Faculty of Veterinary Medicine, University of Lisbon, Avenida da Universidade Técnica, 1300–477 Lisboa, Portugal; University of Iowa Carver College of Medicine, UNITED STATES

## Abstract

In humans, one of the major factors associated with infective endocarditis (IE) is the concurrent presence of periodontal disease (PD). However, in veterinary medicine, the relevance of PD in the evolution of dogs’ endocarditis remains poorly understood. In order to try to establish a correlation between mouth-associated *Enterococcus* spp. and infective endocarditis in dogs, the present study evaluated the presence and diversity of enterococci in the gum and heart of dogs with PD. Samples were collected during necropsy of 32 dogs with PD and visually diagnosed with IE, which died of natural causes or euthanasia. Enterococci were isolated, identified and further characterized by Pulsed-Field Gel Electrophoresis (PFGE); susceptibility to antimicrobial agents and pathogenicity potential was also evaluated. In seven sampled animals, PFGE-patterns, resistance and virulence profiles were found to be identical between mouth and heart enterococci obtained from the same dog, allowing the establishment of an association between enterococcal periodontal disease and endocarditis in dogs. These findings represent a crucial step towards understanding the pathogenesis of PD-driven IE, and constitute a major progress in veterinary medicine.

## Introduction

Infective endocarditis (IE) is an important medical condition in dogs, with high morbidity and mortality rates. Although considered an uncommon disease, with a prevalence ranging from 0.09 to 6.6% [1], its true incidence is undoubtedly underestimated, as its final *in vivo* diagnosis is only possible after echocardiography, by detection of characteristic oscillating vegetative lesions in cardiac valves and valvular insufficiency [1], [2].

In dogs, as well as in humans, IE requires an initial damage of the mitral and aortic valves endothelium, followed by platelet-fibrin deposition and bacterial colonization and adherence [1]. Disease evolution may promote acute congestive heart failure, thromboembolic disease and arrhythmias [1], [3]. IE prognosis depends on the pathogenic profile of associated bacteria, infection severity and affected valves, but it is usually poor. Treatment is only efficient in the early stages of disease and it usually requires the long-term administration of broad-spectrum antibiotics [1].

One major factor related to human IE is the concurrent presence of periodontal disease (PD) [3–6]. In veterinary medicine, this association is considered to be relevant, but research aiming to confirm this link is scarce, most being observational and retrospective [7], [8]. Such studies would be of major importance, as PD is one of the most widespread diseases in dogs, with a prevalence of 44 to 80% [9], [10].

PD has a multifactorial aetiology, depending on several factors, related with the host and the environment [5]. It requires the formation of a plaque, defined as a microbial biofilm in the oral cavity that leads to the inflammation of tooth supporting structures, progressing from a mild gingivitis to severe periodontitis reaching the periodontal ligament and alveolar bone [5], [7], [9]. At this stage, bacteria may disseminate to other organs via bloodstream, causing systemic diseases, including IE [7].

Several bacterial species that colonize humans’ oral cavity have been associated with PD-driven IE, including *Enterococcus* spp. [6], [11–13], also frequently present in the oral cavity of dogs [14]. However, the role of enterococcal PD in IE evolution remains unclear, although this bacterial genus has already been described as the third most common cause of bacterial endocarditis in humans [13], [15].

The present study investigated the possible association between periodontitis and infective endocarditis, by evaluating the presence and genomic relatedness of *Enterococcus* spp. present in the gum and heart of dogs with PD.

## Material and Methods

Swab samples from mitral/tricuspide valves and gums were collected at a private veterinary hospital located in Cascais, Portugal, during the necropsy of 32 dogs (17 males and 14 females, aged between 7 and 17 years) diagnosed with PD. Sampled animals died of natural causes or euthanasia, and were visually diagnosed with IE. Necropsy was performed in a surgically clean room, using adapted surgical techniques, within a maximum of 15 minutes after death [16–18]. All animal work was conducted according to relevant national (DL 113/2013 from 7 August 2013) and international laws (Directive 2010/63/UE).

Swabs were stored at 4°C and transported to the Laboratory of Microbiology and Immunology, Faculty of Veterinary Medicine, University of Lisbon, Portugal, where they were further processed for *Enterococcus* spp. isolation using conventional microbiological procedures [19]. From each sample, up to four typical single colonies presenting distinct morphologies were randomly selected for further characterization. Subsequently, to further confirm the allocation of the isolates as *Enterococcus* spp., PCR amplification was performed according to the method described by Ke *et al*. [20]. Identification at species level was performed by multiplex-PCR using species specific primers and conditions previously described [21] and the genomic relatedness between isolates of the microbial collection was further assessed by *Sma*I-macrorestriction analysis using Pulsed-Field Gel Electrophoresis (PFGE) [22].

Data generated was analysed using the BioNumerics 6.6 software (Applied Maths, Kortrijk, Belgium), which allowed the selection of enterococcal isolates present in both mouth and heart of the same animal; such enterococci were further characterized regarding antibiotic resistance to amoxycillin/clavulanate, ampicillin, chloramphenicol, ciprofloxacin, clindamycin, erythromycin, high-level gentamicin, imipenem, high-level streptomycin, tetracycline and vancomycin [23]. The presence of enterococcal virulence factors was screened by PCR amplification using primers and protocols previously described [24], [25]: genes coding for aggregation substance -agg-, the *E*. *faecalis* antigen A -efaAfs-, the *E*. *faecium* -efaAfm-, the enterococcal surface protein -esp-, the pili-like -ebpABC-, gelatinase -gelE-, cytolysin activator -cylA- and the adhesins of collagen for *E*. *faecalis* -ace- and *E*. *faecium* -acm-. Additionally, plate assays for the evaluation of hemolytic and gelatinolytic phenotypes were also performed [26], as well as screening for biofilm-forming ability using microtiter-plate assays [27], [28].

Reference strains *Enterococcus faecalis* ATCC 29212 and *E*. *faecalis* MMH594 were used as controls, respectively for antimicrobial resistance characterization, and PFGE/virulence studies.

## Results and Discussion

From the 64 samples, 32 from each sampled site, a total of 35 were positive for the presence of *Enterococcus* spp., 21 mouth swabs and 13 from the heart. Overall, 117 enterococci were recovered after bacterial isolation, 99 belonging to the species *E*. *faecalis* and 18 identified as *E*. *faecium*. Subsequently, in order to assess for the genetic relatedness between enterococcal isolates *Sma*I-macrorestriction analysis was performed. For six of the sampled dogs PFGE-patterns observed for enterococci recovered from the mouth were distinct from those obtained from the heart (data not shown), but for seven of the 32 sampled animals PFGE-patterns were identical between mouth and heart enterococci obtained from the same dog (S1 Fig).

Considering that the same isolate was present in both the oral cavity and heart valves of dogs with PD and IE, this suggests the occurrence of enterococci dissemination between the animals’ mouth and heart, as already described in human IE cases [6]. Although the hypothesis of contamination during necropsy or dissemination from intestinal microbiota could be considered, these do not seem possible in our study. As already mentioned, necropsies were performed using proper facilities and techniques, avoiding not only environmental contamination, which would result in a larger number of animals with similar isolates in both gum and heart samples, but also *post-mortem* spread of microorganisms [16–18]. In fact, *post-mortem* spreading from intestines would probably result in changes in the integrity of major organs, which were not observed.

These isolates also presented identical antimicrobial resistance and virulence profiles (Fig 1). Two putative virulence factors previously related with enterococcal endocarditis [15], [29] were observed in all isolates, namely the endocarditis antigen *efaA* and endocarditis and biofilm associated pili *ebpABC*. All isolates also showed the ability to produce biofilm, a major virulence factor related with IE pathogenesis [15]. Other putative virulence traits were also found, but not equally distributed amongst all isolates (Fig 1). All these features are mainly related to bacterial adherence and tissue degradation, crucial steps for IE development and establishment [15], [29], [30]. It is important to refer that this broad distribution of virulence factors amongst *E*. *faecalis* isolated from dogs’ IE cases doesn’t relate to which is observed in humans, since it has been stated that human endocarditis isolates are able to express less virulence determinants than non-endocarditis bacteria [31].

**Fig 1:** *Sma*I-macrorestriction patterns, antimicrobial resistance and virulence profiles of the enterococci clinical isolates. M—mouth, H—heart, TET—tetracycline, S300—high-level streptomycin, E—erythromycin, C- chloramphenicol, CN10—high-level gentamicin, *gelE*–gelatinase coding gene, *efaA*—endocarditis antigen gene, *ebpABC*—endocarditis and biofilm associated pili gene, GEL—gelatinase production, *esp*—enterococcal surface protein gene, *agg*—aggregation substance gene, *ace*—collagen binding protein coding gene, HLY—hemolysin production, *cylA*—cytolysin activator gene.

Regarding dog-associated enterococci antimicrobial resistance profiles (Fig 1), although all isolates were resistant to at least one antibiotic, none was resistant to the most used compounds in veterinary medicine for the treatment of IE promoted by Gram-positive bacteria, which include ß-lactams and quinolones [1]. No multi-drug resistant profiles were observed, but two isolates were resistant to high-level streptomycin and other two were simultaneously resistant to high-level streptomycin and high-level gentamicin, representing a problem due to the possibility of bacterial dissemination to humans, as these compounds represent alternatives for the treatment of *E*. *faecalis* IE in human medicine [13], [15].

## Conclusions

This study allowed us to establish, to our knowledge for the first time, an unquestionable association between periodontal disease and bacterial-endocarditis in dogs. It also outlines the importance of characterizing oral infections caused by uncommon infectious microorganisms, as these can be underestimated and may evolve to severe disease such as IE. Therefore, veterinarians should always advise owners regarding at-home prevention measures for the safeguarding of the oral cavity health of their pets.

## Supporting Information

S1 Fig *Sma*I-macrorestriction patterns, antimicrobial resistance and virulence profiles of the enterococci clinical isolates. (DOCX)
